The article "Biometric Authentication and Correlation Analysis Based on CNN-SRU Hybrid Neural Network Model" was published in 2023. Journal: Comput Intell Neurosci.

# Biometric Authentication and Correlation Analysis Based on CNN-SRU Hybrid Neural Network Model

**DOI:** 10.1155/2023/8389193

**Published:** 2023-03-01

**Authors:** Houding Zhang, Zexian Yang

**Affiliations:** ^1^University of Wollongong, Wollongong, Australia; ^2^China Foreign Affairs University, Beijing, China

## Abstract

With the continuous development of computer technology, many institutions in society have higher requirements for the efficiency and reliability of identification systems. In sectors with a high-security level, the use of traditional key and smart card system has been replaced by the identification system of biometric technology. The use of fingerprint and face recognition in biometric technology is a biometric technology that does not constitute an infringement on the human body and is convenient and reliable. The biometric technology has been continuously improved, and the existing biometric technologies are based on unimodal biometric features. The unimodal biometric technology has its own limitations such as proposing single information and checking data affected by the environment, which makes it difficult for the technology to play its advantages in practical applications. In this paper, we use CNN-SRU deep learning to preprocess a large amount of complex data in the perceptual layer. The data collected in the perceptual layer are first transmitted to CNN convolutional neural network for simple classification and analysis and then arrives at the LSTM session to update again and optimize the screening to improve the biometric performance. The results show that the CNN-LSTM, CNN-GRU, and CNN algorithms show a decreasing trend in accuracy under the three error evaluation criteria of RMSE, MAE, and ME, from 0.35 to 0.07, 0.58 to 0.19, and 0.38 to 0.15, respectively. The recognition rate of multifeature fusion can reach 95.2%; the recognition efficiency of the multibiometric authentication system and accuracy rate has been significantly improved. It provides a strong guarantee for the regional standardization, high integration, generalization, and modularization of multibiometric identification system application products.

## 1. Introduction

The rapid development of computer information technology has put forward higher requirements for the update and processing of information technology [1, 2]. In the field of system security protection, relying solely on hardware devices has been difficult to meet customer needs. The traditional key-based authentication method becomes more and more unreliable and stable due to the large amount of data, the rapid spread, and the simple replication. Therefore, according to customer needs, we provide an overall solution and provide a multibiometric authentication platform to meet their actual needs. Biometric technology is a technology for automatic identification by collecting the physiological characteristics and biological characteristics of the human body [3]. Human biometrics are relatively stable, and there are no problems such as loss and forgetting. Compared with the traditional cryptographic key authentication method [4–7], it has more effective system security. The biometric identification method uses the human body marking method, which is easy to carry with you and can realize real-time collection, identification, and judgment of biometric information. Generally speaking, human biometrics have seven characteristics, including universality, uniqueness, permanence, collectability, acceptability, safety, and performance requirements [8–10]; biometrics do not change with time and the environment. Large changes can be quantitatively collected and analyzed, the collected feature information can meet the needs of users, and the features are not easy to be imitated or forged [11, 12]. The bottom line is that everyone is biometric and different.

The article "Biometric Authentication and Correlation Analysis Based on CNN-SRU Hybrid Neural Network Model" was published in 2023. Journal: Comput Intell Neurosci.

Biometric technology has the characteristics of good anticounterfeiting performance, high security, and reliability and has become the most widely used security and identity authentication technology [13, 14]. Biometric technology relies heavily on physiological or behavioral features, and common face recognition [15, 16], language control [17], and fingerprint recognition [16, 18] can be used as biometrics. At present, the application of the above-mentioned biometric technology has made great progress, and the related scientific research at home and abroad has become more and more extensive. We are conducting a visual analysis of biometrics related to Chinese and English documents in the CNKI database, as shown in Figure 1. We found that the number of studies on biometrics gradually increased from 2000, and after 2005, the number of articles published each year was more than 1000, and in recent years, it reached more than 2000; meanwhile, in the study of the distribution of keywords and topics co-occurring in the articles, we could find that the keywords with the highest frequency were mainly biological characteristics, as shown in Figure 1. Face recognition, fingerprint recognition, algorithm research, recognition technology, etc., show that the algorithm research has gradually deepened and achieved extraordinary results in the research of biometrics. The study [19] focused their work on the application of machine learning to biometric speech, and they focused on the same concept of examining the recognition accuracy of the machine learning algorithm REPTree on a selected speech biometric dataset that was deployed and evaluated with the mining tool WEKA. The goal was to achieve a percentage greater than or equal to 95 in order to accurately classify the given sample data. In terms of processing other biometric information, a systematic study and comparison in ear biometrics has been conducted by [20]. They proposed another idea to perceive the ear in an online irregular orientation. This work can touch on the fitting of inwardly curved ears and the extraction of highlights from the internal drills of the ear edges. Here, the watchful edge recognition computation is used to locate the edges of the ear. The ear images are processed by the shape follower computation and then the rough images with edges are found as the yield of the frame. Finally, each of the three component vectors is decontrasted and compared with an alternate library of ear pictures and tracked for a specific match. In [21], they mainly used algorithms to enhance the security of face recognition techniques. In their paper, they proposed a fast and robust fuzzy C-mean clustering (FRFCM) algorithm and face recognition optically selective encryption scheme for biometric medical images. In the proposed scheme, a new selection method for obtaining regions of interest (ROI) based on the FRFCM algorithm is proposed. The security and robustness of the proposed cryptosystem is also verified by numerical simulations. The study [22] systematically analyzes the key points and difficulties of biometric techniques in spectral imaging. The reliability of conventional face recognition systems working in the visible range will be affected by light variations, pose variations, and spoofing attacks. There are no large databases available for benchmark evaluation. Existing databases do not capture the same test subjects on all possible frequency bands for which experimental evaluations have been carried out. Also, this has been limited so far due to the small number of test objects and their images in the existing database. Deep learning based methods require a large number of parameters for training. This leads to overfitting due to the small number of such samples in the existing databases. The study [12] was conducted to remotely determine current human biological parameters by algorithmically processing infrared images of human faces. The problems that hinder the widespread use of remote biometric algorithms in practice are highlighted. The urgency of creating a metrological database containing video recordings of face images in the infrared range to assess the efficiency of biometric algorithms, time-synchronized records of human biometric parameters, and information on the complexity of the test tasks performed was confirmed. The structure of the laboratory system used to acquire complex data of the tested person is considered. A typical data structure for a single test cycle is given as shown in Figures 1 and 2.

The article "Biometric Authentication and Correlation Analysis Based on CNN-SRU Hybrid Neural Network Model" was published in 2023. Journal: Comput Intell Neurosci.

Through the analysis and summary of the above-given literature research work, it can be seen that the development and application optimization of deep learning in biometrics has carried out systematic excellence. However, the research work on multibiometrics technology is still at an immature stage, and the evaluation standards are not uniform. Secondly, multibiometrics authentication also increases the burden on users. Not perfect in multibiometric fusion. Therefore, this paper studies the multibiometric recognition system through the fusion of facial features, speech recognition, and fingerprint recognition. In addition, we introduce three algorithms of CNN, LSTM, and GRU to extract and fuse biometric parameters. Optimization studies are conducted. In view of the problems such as the continuous increase of biometric data, the untimely update of features, and the resulting system lag, we optimize the algorithm to improve the system update rate and improve the security and stability of the biometric identification system. In addition, we analyze and study the collected 2000 data, and verify the robustness and accuracy of the algorithm through simulation.

Biometric identification technology, referred to as biometrics, is the identification and authentication of personal identity by acquiring biometric characteristics unique to human beings. We classify these inherent biometric characteristics into two major categories, namely, physiological characteristics and behavioral characteristics. Physiological characteristics are those that are innate and would not have led to changes in the absence of special factors. Typical examples are fingerprints, iris, DNA, etc. The other behavioral traits are mainly acquired habits. Typically, they are the voice of the person speaking, the font of the signature, etc., [23, 24].

All biometrics include the following processes: acquisition, decoding, comparison, and matching. The basic process is shown in Figure 3.

Biometric identification technology is mainly through the detection of the physical characteristics that the human body has always had so as to carry out identity confirmation, not all the characteristics of the human body can be used as the collection point for identification, and the characteristics that need to meet the following conditions can be used as the identification target:

1. Uniqueness
2. Most of the human body's biological information has the characteristic of uniqueness, uniqueness mainly for the comparison between individual people, absolutely unique. In the case of fingerprints, the texture details are not the same between each individual.
3. Stability
4. The biological information of a human individual always remains the same from birth to death, but of course, if the feature is changed or damaged by human or external factors, it will change. For this reason, it can be used to identify individuals.
5. Identifiability
6. The biometric characteristics of human beings are very different from each other, and by using certain computer algorithms, it is possible to distinguish this information and identify the key elements of the characteristics, making it possible to use the identification technology in a wide area.
7. Capturability
8. With the development of computer technology and related hardware technology, the image quality and pixels of the feature image information collected by the instrument are also improved, making the image a convenient carrier for recognition.

The article "Biometric Authentication and Correlation Analysis Based on CNN-SRU Hybrid Neural Network Model" was published in 2023. Journal: Comput Intell Neurosci.

## 2. The Feasibility of CNN Network in Biometric Authentication

With the rapid development of science and technology, more and more information is obtained and authorized remotely through online, and the required resources can be legally accessed and the right of application is a necessary condition for the security of the internal data of the communication system. In addition, in the network environment, how to identify and verify the reliability of biometric information, safely realize remote authentication, and ensure the privacy of biometrics from illegal use has become the main problem to be solved in this paper. Therefore, this paper proposes a 2D CNN network to track the lines in electronic data and implement vectorization to realize the recognition processing. 2D CNN can not only extract features from a large number of graphs, data reconstruction, and other preprocessing methods. At the same time, each computing layer itself has the same weight for sharing links, which greatly reduces the computing cost and computing time and avoids too many parameters affecting the clarity of text/graphics. In addition, LSTM can easily and accurately capture the main information of the sequence from pictures to speech because of its linear structure. Strive to propose a CNN-LSTM network based on deep learning biometric authentication to provide an effective solution quickly, conveniently, and safely.

### 2.1. Structure of CNN Network

Figure 4 presents a generalized framework for digital image source forensics under the CNN model theory. In the image preprocessing, the image to be detected is first cut into image blocks (*P*_*k*_ in Figure 4(a) indicates the *k* th image block), and then the image fingerprint characterizing the source of the shot is extracted using CNN (image feature extraction in Figure 4(b)), and the detection result *Y*_*k*_ of each image block is output (*Y*_*k*_ in Figure 4(c) indicates the feature extractor predicts the label for the *k* th image block), and the majority voting algorithm is used to fuse the detection results of the *k* th image block and output the image level prediction results, i.e., device model multiclassification identification.

The article "Biometric Authentication and Correlation Analysis Based on CNN-SRU Hybrid Neural Network Model" was published in 2023. Journal: Comput Intell Neurosci.

### 2.2. Learning Algorithm of CNN Network

The training process of the CNN network is mainly divided into forward propagation and back propagation [25]. First, by inputting data to the convolution layer, the feature extraction is performed on the convolution operation based on the filter and the convolution kernel (Kernel), the feature map is obtained, and the bias term is added to it, and then the activation function (ReLu, Tanh, sigmoid, and softmax) to calculate the output of the convolutional layer; the pooling layer samples the data processed by the receiving convolutional layer, and then converts the feature map into a vector by stretching and sums the weighted biases. Finally, the class probability output is obtained through the activation function, and the calculation is repeated until the loss function is the minimum value [26].

(1) Calculation of the convolutional layer. The convolution formula is shown in equation (1), the input *x* is weighted *w*, and the bias *b* is added, and finally the total sum obtained is output through the nonlinear activation function *f*.
  (1) $$\begin{array}{c} a_{d,i,j}=f\left(\overset{D-1}{\underset{d=0}{\sum }}\overset{F-1}{\underset{m=0}{\sum }}\overset{F-1}{\underset{n=0}{\sum }}w_{d,m,n}x_{d,j+m,j+n}+b\right)\text{.} \end{array}$$
Among them, *D* and *F* are the number of filters and the size of the convolution kernel, respectively.
(2) Calculation of pooling layer and full connection. The pooling layer retains the main effective information by locally sampling the feature map and reduces the influence of unnecessary data on the calculation result. In addition, as long as there is a relative relationship with the main information of the feature map, no matter whether the image is scaled, distorted, translated, etc., the accuracy of the result cannot be affected. After the data is passed through the pooling layer, a large number of parameters can be filtered out, which can improve the training accuracy and reduce the error. The average sampling method sampled in this paper samples the feature map, and in the traversed region, the average value is selected as the new feature of the region. Due to the characteristics of CNN itself, under the action of the fully connected layer, the output of the convolutional layer is weighted w offset summation, and then output through the activation function *f*, as shown in the following equation:
  (2) $$\begin{array}{c} y=f\left(w\cdot x+b\right)\text{.} \end{array}$$
(3) Calculation of softmax output layer. The activation function nonlinearizes the total number of weighted bias sums to solve the multiclass problem, and its calculation formula is as follows:
  (3) $$\begin{array}{c} y_{k}=\frac{e^{a_{j}}}{\overset{n}{\underset{i=1}{\sum }}e^{a_{i}}}\text{.} \end{array}$$
In the formula, *n* is the number of inputs.
(4) Back propagation
(1)–(3) are forward propagation, and the error is calculated by the loss function for reverse propagation. The process is divided into three main parts:
  (a) Calculate the network error from the predicted and actual results:
    (4) $$\begin{array}{c} \delta^{i,l}=-\;\left(y_{\text{real}}\left(i\right)-y_{\text{predict}}\left(i\right)\right)*\sigma \left(a^{i,l}\right)\text{.} \end{array}$$
  Among them, *y*_predict_ is the prediction data, *y*_real_ is the experimental data.
  (b) The calculation error is passed in the reverse direction. The specific propagation formula of CNN is as follows:
  Fully connected layer.
    (5) $$\begin{array}{c} \delta^{i,l}={\left(w^{l+1}\right)}^{T}\delta^{i,l+1}⊙\sigma \left(a^{i,l}\right)\text{.} \end{array}$$
  Convolutional layer.
    (6) $$\begin{array}{c} \delta^{i,l}=\delta^{i,l+1}*rot180\left(w^{l+1}\right)⊙\sigma \left(a^{i,l}\right)\text{.} \end{array}$$
  Pooling layer.
    (7) $$\begin{array}{c} \delta^{i,l}=\text{upsample}\left(\delta^{i,l+1}\right)⊙\sigma \left(a^{i,l}\right)\text{.} \end{array}$$
  Among them, *l* is the current layer and *σ*(*a*^*i*,*l*^) is the activation function.
  (c) The final goal of reverse transfer is to update the weight *w* and bias *b*, and the specific calculation is as follows.
  Weight update in the fully connected layer:
    (8) $$\begin{array}{c} w^{l}=w^{l}-\alpha \overset{m}{\underset{i=1}{\sum }}\delta^{i,l}{\left(\alpha^{i,l-1}\right)}^{T}\text{.} \end{array}$$
  Fully connected layer bias update.
    (9) $$\begin{array}{c} b^{l}=b^{l}-\alpha \overset{m}{\underset{i=1}{\sum }}\delta^{i,l}\text{.} \end{array}$$
  Weight update in the fully connected layer.
    (10) $$\begin{array}{c} w^{l}=w^{l}-\alpha \overset{m}{\underset{i=1}{\sum }}\alpha^{i,l-1}*\delta^{i,l}\text{.} \end{array}$$
  Bias update in fully connected layer:
    (11) $$\begin{array}{c} b^{l}=b^{l}-\alpha \overset{m}{\underset{i=1}{\sum }}\underset{u,v}{\sum }{\left(\delta^{i,l}\right)}_{u,v}\text{.} \end{array}$$

Among them, *α*^*i*,*l*−1^ is the output of the ith neuron in the *l*-1th layer.

The article "Biometric Authentication and Correlation Analysis Based on CNN-SRU Hybrid Neural Network Model" was published in 2023. Journal: Comput Intell Neurosci.

In addition, this paper chooses the cross entropy loss function as the loss function, and the formula is as follows:

(12) $$\begin{array}{c} J_{c}=-\frac{1}{N}\overset{N}{\underset{1}{\sum }}\overset{k}{\underset{i=1}{\sum }}y\left(i\right)\log\;\left(y_{c}\left(i\right)\right)\text{.} \end{array}$$

Among them, *y*_*c*_(*i*) is the predicted value, *y*(*i*) is the real value, and *N* is the number of samples.

### 2.3. LSTM Network

A single-channelLSTM-based method for analyzing factors related to youth physical activity behavior mainly includes: LSTM neural networks that use memory units to avoid gradient disappearance and gradient explosion during backpropagation and can learn long-term dependencies and make full use of historical information. The LSTM was improved and extended in 2013 by [27, 28], making it widely used in natural language processing, speech recognition, and other fields.

As shown in Figure 5, the LSTM unit has a memory unit *c* for saving historical information. The updating and utilization of the history information is controlled by three gates: input gate *i*, forget gate *f*, and output gate *o*. The updating process of the LSTM unit at time *t* is as follows:

(13) $$\begin{array}{c} i_{t}=\left.\sigma W_{i}x_{t}+U_{i}h_{t-1}+V_{i}c_{t-1}\right)\text{,}\\ c_{t}=\tan\;h\left(W_{c}x_{t}+U_{c}h_{t-1}\right)\text{,}\\ f_{t}=\left.\sigma W_{f}x_{t}+U_{f}h_{t-1}+V_{f}c_{t-1}\right)\text{,}\\ c_{t}=f_{t}⊙c_{t-1}+i_{t}⊙c_{t}\text{,}\\ o_{t}=\left.\sigma W_{o}x_{t}+U_{o}h_{t-1}+V_{o}c_{t}\right)\text{,}\\ h_{t}=o_{t}⊙\tanh\left(c_{t}\right)\text{,} \end{array}$$

where *x*_*i*_ is the input data of the memory unit, *σ* is the logistic sigmoid function, the symbol ⊙ is the dot product operation between vectors, and *W*_*i*_, *W*_*f*,_*W*_*c*_, *W*_*o*_, *U*_*i*_, *U*_*f*_, *U*_*c*_, *U*_*o*_, *V*_*o*_ is the weight matrix. *i*_*t*_, *o*_*t*_, *f*_*t*_, *c*_*t*_ are the values of the input gate, output gate, forgetting gate, and memory cell at time *t*, respectively, *c*_*t*_ are the values of the candidate memory states of the memory cell, and *h*_*t*_ are the outputs of the LSTM cell at time *t*.

For the analysis of the factors associated with youth physical activity behavior, we first used the random undersampling method to obtain a balanced sample of the factors associated with each youth physical activity behavior and then used a single-channel LSTM neural network as the classification method.  Figure 6 shows the framework of the single-channel LSTM neural network classifier, which has only one LSTM layer. The first dashed box shows the internal structure of the single-channel LSTM model, and the second dashed box shows the process of unbalanced samples. The input to the LSTM model is a word vector representation of the training samples, which has good semantic features and is a common way to represent word features. The input feature vectors are passed through the LSTM layer to obtain high-dimensional vectors, which can learn deeper features that can better describe the samples. The fully-connected layer is similar to the hidden layer of a traditional multilayer perceptron, receiving all the outputs from the previous layer, weighting and summing these output vectors, and propagating the weighted outputs through the excitation function to the dropout layer. In this experiment, the layer uses ReLu as the excitation function, which reduces the interdependence between parameters and is closer to the biological activation model, and the excitation function is shown in (14).

(14) $$\begin{array}{c} g\left(x\right)=\max\;\left(0,x\right)\text{,} \end{array}$$

where *x* is the output vector and the ReLu function sets all values less than 0 to 0, with the ability to bootstrap moderate sparsity. The dropout layer randomly leaves some hidden layer nodes in the network inactive during training and prediction, reducing the number of features and effectively preventing the network from overfitting. The dropout layer appears as a hidden layer in the LST M neural network model, as shown in the following equation:

(15) $$\begin{array}{c} g=h^{*}•D\left(p\right)\text{,} \end{array}$$

where *D* denotes the dropout operator and *p* is an adjustable superparameter (the ratio of retained hidden layer cells).

The article "Biometric Authentication and Correlation Analysis Based on CNN-SRU Hybrid Neural Network Model" was published in 2023. Journal: Comput Intell Neurosci.

Finally, the output of the single-channel LST M model is used to classify the samples by the Softmax output layer. We choose the category with the highest posterior probability as the prediction label, as shown in the following equation:

(16) $$\begin{array}{c} {\text{label}}_{\text{pred}}={\mathrm{argmax}}_{i}P\left(\left.Y=i\right|x,W,U,V\right)\text{,} \end{array}$$

where *x* is the upper layer output vector, *i* is the label prediction, *W*, *U*, *V* are the coefficient matrices in the LSTM update method, and label_pred_ is the predicted label with the highest posterior probability.

### 2.4. Data Preprocessing and Model Parameter Determination

#### 2.4.1. Normalization Processing

Since the magnitude of data input by different channels is very different, it will affect the increase of training error. Therefore, we first need to normalize the data to normalize all inputs to the same interval. In this paper, we choose max-min normalization for normalization, and the calculation method is as follows:

(17) $$\begin{array}{c} X=\frac{x-x_{\min}}{x_{\max}-x_{\min}}\text{.} \end{array}$$

Among them, *x*_max_ is the maximum value in the data set, *x*_min_ is the minimum value in the data set. After normalization, the training error will not increase due to the order of magnitude between the data.

The article "Biometric Authentication and Correlation Analysis Based on CNN-SRU Hybrid Neural Network Model" was published in 2023. Journal: Comput Intell Neurosci.

#### 2.4.2. Determination of Model Parameters

The main influencing factors of biometric vectorization are physiological characteristics and behavioral characteristics. Physiological features include fingerprints, facial images, and irises which are identified according to each individual's unique biological features; behavioral features are gait, voice, handwriting, etc., which are also a method of identifying the appraiser. For example, when identifying a person's handwriting, the outline of the font is clear and distinct, and the effect of the network calculation on displaying the vector diagram is more obvious; the more the number of words, the more data the network can obtain, which makes the network output results have a certain robustness. Specific steps are as follows:

1. The two categories of parameters, physiological characteristics, and behavioral characteristics, are used as the input nodes of the prediction model, and predictions are used as the output nodes of the prediction model.
2. The hidden layer plays a key role in the network architecture. The number of filters in the convolutional layer in this model 2D CNN is 2, the size of the convolution kernel is 16, the stride is 1, and the padding is 2. The LSTM layer nodes are 4, and the fully connected layer nodes are 3.
3. In order to adjust the appropriate learning rate parameters and avoid overfitting or underfitting, it is necessary to continuously test and adjust. The Adam algorithm model is used, and the learning rate parameter is finally selected as 0.0014 and the decay rate is 0.08 [29].
4. After data preprocessing, the data can be used as an input layer node to output the results.

#### 2.4.3. Several Multibiometric Systems

We can use different feature points, sensors, and feature extraction quantities and methods, multibiometric systems can have the following combinations:

1. Unimodal biometric, a combination of multiple sensors, where the biometric features of the same target are acquired by multiple sensors, so that the sample data can be acquired twice. By acquiring face feature data in this way, this data is combined in the data layer and the matching layer, which can effectively improve the recognition rate of the face recognition system.
2. The combination of unimodal biometric features, multiple classifiers, and one sensor is different from unimodal biometric features in that biometric data is acquired by one sensor and these sample data are processed by multiple classifiers. The respective defined features are generated. Matching at the logical layer can improve the recognition rate.
3. Unimodal biometric features, a combination of multiple categories, in the case of iris and fingerprint features, extracts two or more biometric information from the target person. This combination does not require multiple sensors to acquire information and is not particularly demanding for multiple feature extraction and matching models.
4. Combination of multiple biometric features, the combination is to use multiple biometric features for recognition and obtain different feature data by different sensors. Due to the relative independence of the biometric features and thus the accuracy of the recognition system is greatly improved.

The article "Biometric Authentication and Correlation Analysis Based on CNN-SRU Hybrid Neural Network Model" was published in 2023. Journal: Comput Intell Neurosci.

## 3. Experimental Verification and Comparative Analysis

### 3.1. Comparative Analysis of Recognition Accuracy of Biometric Results

In order to verify that the CNN-LSTM network has better performance, this paper compares and analyzes CNN, CNN-GRU, and CNN-LSTM. In order to further analyze the performance of these three networks, we choose root mean square error as the evaluation index: root mean square error (RMSE): measure the error between the observed value and the actual value which is calculated as follows:

(18) $$\begin{array}{c} RMSE\left(X,h\right)=\sqrt{\frac{1}{N}\overset{N}{\underset{i=1}{\sum }}{\left(h\left(x_{i}\right)-y_{i}\right)}^{2}}\text{.} \end{array}$$

Specifically, compared with the actual results, the RMSE of the CNN-LSTM algorithm is smaller than that of the CNN-GRU algorithm and CNN algorithm, which are 0.07, 0.17, and 0.35, respectively, and the CNN-LSTM algorithm is improved by 59% and 80%, as shown in Figure 7. Using the CNN-LSTM recognition technology with fast acquisition speed and high efficiency of feature comparison for effective recognition has great potential value for future biometric optimization, as shown in Figure 7.

In addition, the error of the CNN-LSTM algorithm is smaller than that of the CNN-GRU algorithm and CNN algorithm, which are 0.19, 0.31, and 0.58, respectively, and the CNN-LSTM algorithm improves 38% and 57% compared with the actual results of physiological features, as shown in Figure 8.

Finally, compared with the actual results, the CNN-LSTM algorithm has smaller errors than the CNN-GRU algorithm and CNN algorithm in terms of physiological and behavioral features of speech, which are 0.15, 0.22, and 0.38, respectively, and the improvement of the CNN-LSTM algorithm is 32% and 60%, respectively, illustrating the excellent performance of CNN-LSTM deep learning in biometric recognition as shown in Figure 9.

The article "Biometric Authentication and Correlation Analysis Based on CNN-SRU Hybrid Neural Network Model" was published in 2023. Journal: Comput Intell Neurosci.

In the biometric system, only the sound feature is used in long-term applications, and the biometric recognition accuracy can reach up to 67.7%, the fingerprint recognition accuracy can reach up to 82.1%, and the face recognition accuracy can reach up to 84.5%. The multifeature fusion recognition can reach up to 95.2%. This shows that the algorithm can better match the actual needs of biometric identification. It can greatly improve the recognition accuracy and improve the recognition efficiency as shown in Figure 10 and Table 1.

## 4. Conclusion

In this paper, we give a basic description of the concept of multicommunication framework and neural network algorithm and introduce the structure and calculation process of SRU algorithm for wireless communication receiving module. And, we compared the three algorithms of SRU, GRU, and LSTM, and the hidden layer, number of nodes, number of iterations, learning rate, and activation function in the network structure are all the same. the result shows the following theories:

1. In the fingerprint biometric identification of physiological characteristics, the accuracy of CNN-LSTM, CNN-GRU, and CNN algorithm shows a downward trend under the RMSE error evaluation standard, from a maximum of 0.35 to 0.07, a maximum increase of 80%;
2. The accuracy of CNN-LSTM, CNN-GRU, and CNN algorithms in facial biometric recognition in physiological features shows a downward trend under the RMSE error evaluation standard, from a maximum of 0.58 to 0.19, a maximum increase of 57%;
3. In the biometric recognition of sounds in behavioral features, the accuracy of CNN-LSTM, CNN-GRU, and CNN algorithms shows a downward trend under the RMSE error evaluation standard, from a maximum of 0.38 to 0.15, a maximum increase of 60%; It illustrates the excellent performance of CNN-LSTM deep learning in biometric identification.
4. Multifeature fusion recognition can reach up to 95.2%, compared with 84.5%, 82.1%, and 67.7% of single face recognition, fingerprint recognition, voice recognition, etc., which have a great improvement, which shows that the algorithm can better match the actual needs of biometrics. It provides a strong guarantee for the regional standardization, high integration, generalization, and modularization of multibiometrics system application products.

At present, the system has been applied in a large number of customers, but after the actual use, the system still reveals some problems, and recognition technology still needs to be improved; these will be the focus of later work. With the biometric identification technology application in the field is deepening and the scope is expanding, many enterprises are investing more and more in this technology. The updated speed of biometric identification technology will also be accelerated. For the application software of biometrics technology, if it needs to have a lasting vitality, it needs to keep up with the advanced technology. Due to the development period and resources, this system still has many unsatisfactory points and needs to be improved later.

The article "Biometric Authentication and Correlation Analysis Based on CNN-SRU Hybrid Neural Network Model" was published in 2023. Journal: Comput Intell Neurosci.

## Figures and Tables

**Figure 1:** Trends in biometrics research.

**Figure 2:** Proportion of research on keywords and topics.

**Figure 3:** Biometric basic processing flow.

**Figure 4:** Digital image source framework based on CNN. (a) Image preprocessing. (b) Image feature extraction. (c) Classification result voting.

**Figure 5:** LSTM unit.

**Figure 6:** Single-channel LSTM neural network classifier framework.

**Figure 7:** RMSE error plot of fingerprint biometrics in physiological features.

**Figure 8:** RMSE error plot of face biometric recognition in physiological features.

**Figure 9:** RMSE error plot for biometric recognition of voices in behavioral traits.

**Figure 10:** Overall recognition result of biometric identification of fingerprints, faces in physiological features, and voices in behavioral features.

**Table 1:** Comparison of RMSE of three algorithms in different application scenarios.

	Fingerprint identification	Image recognition	Voice recognition
CNN	0.35	0.58	0.38
CNN-GRU	0.17	0.31	0.22
CNN-LSTM	0.07	0.19	0.15

## Data Availability

The experimental data used to support the findings of this study are available from the corresponding author upon request.
